This article has been retracted.

# Study of the synergistic effect of analogical and explicit learning in beginning junior tennis players

**DOI:** 10.1016/j.heliyon.2024.e38590

**Published:** 2024-09-27

**Authors:** Jiyan Xu, Weiwei Xu, Mengjiao Sang

**Affiliations:** a Capital University of Physical Education and Sports, Beijing, China; b Beijing University of Chemical Technology, Beijing, China; c Shandong University, Jinan, Shandong, China

**Keywords:** Junior tennis for beginners, Analogical learning, Explicit learning, Synergistic effects

## Abstract

Motor skill learning is a field where implicit and explicit synergistic learning is particularly evident in authentic situations. While current research on analogical learning, an effective method of implicit learning, is largely focused on theoretical discussions and separability studies, there are relatively few studies that combine analogical learning with explicit learning. In this study, a one-way experimental design was utilized to investigate the synergistic effect of analogical learning and explicit learning on the acquisition of forehand hitting skills in beginning tennis players. A total of thirty-nine children aged 6–8 years were randomly assigned to different groups: one group learned through analogical learning after explicit learning, another group learned through analogical learning followed by explicit learning, and the final group learned through alternating analogical and explicit learning. The performance of each group was evaluated based on retention and transfer tests, measuring batting accuracy, action scores, and number of knowledge mastery. The results showed that the group that underwent analogical learning followed by explicit learning performed better compared to the other two groups. These findings provide theoretical support and practical guidance for the learning of tennis skills of children beginners and the teaching of coaches.

## Highlights

• Different combinations of analogical and explicit learning can affect motor skill learning.
• Beginning junior tennis players were researched combining analogical and explicit learning.
• The analogical-explicit combination may be beneficial for the development of general motor programs in young beginners.

## 1 Introduction

Implicit and explicit learning are the two fundamental styles of motor skill acquisition [1]. Compared to relying solely on implicit or explicit learning, combining the two can produce better performance, and this positive impact has been proven [2,3]. Explicit learning refers to purposeful, conscious learning that necessitates conscious effort [4]. Implicit learning, the ability to unconsciously acquire structured rules in the environment, is an important mechanism for early childhood learning of language, motor and social skills [5]. Analogical learning is a new method of implicit learning, which is the process of comparing two or two types of things to find out their similar relationship at a certain level of abstraction, and using this as a basis for transferring and generalizing knowledge about one type of thing to another, so as to acquire or understand new knowledge [6,7]. Analogical learning modeling is a common method of analogical learning, in which conceptual goals and concepts are analogized to identify characteristics of both and draw conclusions [8]. Analogical learning allows learners to acquire skills on a less linguistic basis through motor metaphors, i.e., the use of imagery and concrete signals can help learners understand motor skills, reduce reliance on cognitive resources, and accelerate the acquisition of motor skills [9]. Analogical learning reduces the reliance on linguistic information in motor skill learning, and the metaphors is intuitive, interesting, and widely used in sports [10]. Children have weaker cognitive abilities, with limited capacities for storing and manipulating information, and the dominance of the first signal system. Analogy learning can use image-specific signals to reduce conscious processing and alleviate working memory load [11]. Some scholars have found experimentally that analogical learning is more likely to maintain the stability of motor performance than explicit learning in the presence of stress [12], and analogical learning is significantly less affected by stress than explicit learning [13]. In this study, explicit learning involves providing direct and concrete language guidance on body and limb movements, while analogical learning involves guiding students in learning tennis skills using analogical language (i.e., metaphors).

As a special group of children, their cognitive deficiencies make it difficult to use specific verbal instructions to understand and master motor skills, so a large number of experiments have been conducted to explore ways to help children quickly master tennis skills. Some studies have found that visual and tactile signals have a good role in promoting the learning of children's tennis skills [14], and auditory can also play an auxiliary role in the process of learning tennis skills [15]. In multimedia teaching, the image signals can increase the enthusiasm and interest of children, and improve the effect of children learning tennis skills [16]. In addition, by exploring the effects of internal and external attentional focus instruction on children's tennis skills, it was found that both external and internal attentional focus helped children learn tennis forehand and backhand skills, and external attentional focus was more effective than internal [17]. Analogical learning and explicit learning have been studied more extensively in other motor skills, but there are fewer studies in tennis, and most of them are separated experimental studies, which mainly verified that analogical learning has the characteristics of implicit learning, while studies on the synergistic effect of the two are rare.

The International Tennis Federation (ITF) launched the Tennis Play&Stay program in 2007, and China launched the “Little Tennis” project in 2023, both of which aim to promote the learning and development of children's tennis skills. In addition, many famous tennis players such as Federer, Djokovic and so on began to contact with tennis training at the age of 4–6 years old, so it can be seen that the cultivation of children's tennis beginners in the early stage plays an important role in the connection with the professional training in the later stage. The cognitive ability of children beginners has certain specificity. In the complex process of motor skill learning, analogical learning helps children to quickly master basic motor skills, and explicit learning helps to strengthen the details of the movement. However, the timing of the two, and the most optimal combination of the two and the effect is not clear. In order to investigate the effects of three different combinations of analogical learning followed by explicit learning, explicit learning followed by analogical learning, and alternating analogical learning and explicit learning on the learning efficiency of tennis skills of children beginners, the present study adopted a one-way experimental design and randomly divides 39 children beginners aged 6–8 years old into three groups, aiming at exploring the optimal combination and their effects, so as to provide theoretical support for children to better master the tennis forehand and improve the learning efficiency of children's sports skills.

## 2 Objects and research methodology of the study

### 2.1 Objects of the study

This study involved children aged 6–8 years who were beginners of tennis at a tennis club located in Haidian District, Beijing, China. All participants were novice learners in tennis skills for the first time and had not previously studied similar sports such as badminton, table tennis, volleyball, or others. A total of 39 children were recruited and randomly assigned to three groups: explicit-analogical group (explicit learning followed by analogical learning), analogical-explicit group (analogical learning followed by explicit learning), and alternation group (alternation between explicit and analogical learning). Each group included 13 children. The average age and standard deviation of the participants in the explicit-analogical group, analogical-explicit group, and alternation group were 7.00 ± 0.82, 6.92 ± 0.86, and 6.92 ± 0.76, respectively.

### 2.2 Ethical approval

This study was approved and obtained the proof of Ethics WAIVER from the College of Humanities and Law, Beijing University of Chemical Technology, China on August 27, 2023. Written informed consent was obtained from the legal guardians of all the participants and assent was also obtained from every participant. The content of this experiment will not cause any adverse consequences, nor will it have any negative impact on the physical and mental health, learning, and daily life of children.

### 2.3 Research methodology of the study

#### 2.3.1 Research design

There were 3 levels of within-subject factors (learning styles): explicit-analogical learning, analogical-explicit learning, and alternation learning. In terms of the experimental design cycle in related studies, the average duration is around one week [9,11,18]. The experimental content selected in this study focused on learning tennis forehand skills among children. The difficulty level of the content, the age of the subjects, and their foundation are similar to those in such studies. Therefore, the experimental period for this study is set at 10 days, and it is expected to produce experimental effects.

#### 2.3.2 Experimental control

Thirteen identical rackets were prepared, and the same racket was used for all three groups during both the learning and testing sessions, which were conducted in daylight to minimize the influence of lighting conditions. The three groups were taught in different combinations, but every effort was made to ensure that each child received an equal amount of teaching time and executed the same number of strokes during each session. Tests were conducted when the subjects were in their best possible condition and the results were averaged across the two groups to reduce the effects of lighting. The two sets of tests were averaged to minimize errors. Pressure mainly stems from teaching expectations and tasks [13], and analogical and explicit teaching experience different levels of pressure. In this study, the pressure factor was controlled using practice time, with all three groups receiving consistent explicit instruction time. The main objective of the experiment was to observe which group performs better under consistent pressure conditions across the three groups. Every effort was made to control irrelevant variables in order to enhance the accuracy of the data.

#### 2.3.3 Experimental tasks

The children were instructed to learn and practice the proper technique of a tennis forehand stroke. As shown in Fig. 1, the subject holds the racket and stands at the midpoint of the baseline, denoted as point T, while the experimenter is positioned in front and to the right at point K (primarily for right-handed forehand learners), extending the arm vertically to drop the ball. C1 and C2 represent the positions of two cameras. Point K serves as the ball toss point for the pre-test and retention test, while point E is the ball toss point for the transfer test, with the green shaded area indicating the ball toss region for the transfer test. The subject hits the ball forehand for scoring in as many of the highest-scoring areas as possible, with 1, 2, and 3 representing different scoring regions. Before the practice session, it was important to inform the participants that this study focused on improving hitting accuracy and maintaining a standardized posture, rather than emphasizing hitting speed in order to avoid compromising the balance between speed and accuracy.

**Fig. 1:** Schematic plan and scoring areas.

#### 2.3.4 Learning guideline

The forehand stroke can be broken down into five distinct parts: the preparation posture, the backswing posture, the lowering posture, the swing posture, and the follow-through posture. Each of these parts necessitates specific explicit and analogical instructions, as illustrated in Table 1. Three groups underwent training in a different sequence. In the experiment, explicit instructions are longer and more complex compared to analogical instructions. Therefore, with the total training time being equal, the explicit instruction time is longer than the analogical instruction time. Questioning was used to ensure that the subjects understood and mastered the instruction phrases and movements.

**Table 1:** Instructions of each part of the forehand stroke.

Movement entry	Explicit learning guides	Analogical learning guides
Preparation posture	1 Face the net with your feet just far enough apart to drop the head of a racket. 2 Bend your knees slightly and lower your center of gravity. 3 Make small steps ready to hit the ball. 4 Left hand on racket, head at eye level, eyes on ball.	1 It's like getting ready to jump in heels.
Backswing posture	5 Turn your right foot as if it were the stationary leg of a circle gauge. 6 The body rushes to the side. 7 Racket stands behind you, don't pinch your arm, arm slightly bent.	2 Turn your body and hide the racket behind your back.
Lowering posture	8 Lower the head of the racket to the level of the ground.	3 Imagine a puppy next to you and gently tap it on the head with a paddle.
Swing posture	9 Turn and hit the ball. Shift your weight forward onto your left foot. 10 Turn your body to the left and at the same time push out the racket with your right arm from the lower right to the front left. 11 Hit the ball with the racket face perpendicular to the ground, don't press down on the racket face.	4 Imagine your body as a circular gauge, rotating on the axis of your right foot. 5 Throw the racket like a whip.
Follow-through posture	12 After hitting the ball, swing the racket to the top of the back of the left shoulder and raise the elbow to the front of the mouth. 13 Wrist to the side of the left ear. 14 Handle and elbow pointing forward. 15 Lift your right heel and punch to your right rear.	6 Imagine throwing a sack over your left shoulder, i.e., the action of carrying a sack, with the elbow blocking the eyes.

#### 2.3.5 Experimental procedure

The experimental period lasted for 10 days with two modules, with each day consisting of 1.5 h of training in the same manner and number of exercises. On the first day, after warm-up activities and instruction on the forehand batting grip, the pre-test was conducted with each subject performing 20 strokes. Following this, Module 1 practice began. Before the practice, the experimenter demonstrated the movement once centrally and provided corresponding instructions. Subjects then swung the racket 20 times as a group and proceeded to individually practice hitting the ball 20 times. While one subject hit the ball, an assistant organized the other subjects to juggle the ball behind a curtain, thus preventing observation and experiential learning. On the sixth day, the training moved on to Module 2. On the tenth day, after a 10-min break, a retention test was conducted with the subjects performing 20 forehand strokes. Subsequently, a transfer test was conducted. In this test, subjects stood in the same position while the experimenter randomly threw the ball by hand at the junction of the serving line and the singles sideline. Subjects were then required to hit the ball into the scoring area. No instructions were given by the experimenter during the testing phase. Subjects were verbally instructed during the exercises and asked to dictate their knowledge of the movements, and the support staff and the experimenter observed their completion to ensure that they understood and mastered the exercises.

A retention test is a test administered after a period of rest following practice, where the subject may have a memory of the previously practiced skill and a retention of the movement in the motor skill area. On the other hand, the transfer test was conducted after a longer period of time since the practice session, and subjects may have forgotten the technical sessions. Both tests had similar objectives in terms of evaluating skill retention over time. However, the key distinction lies in the fact that the retention tests were conducted under identical tasks and conditions, while the transfer tests allowed for variations in tasks and conditions. In the retention test, the experimenter threw the ball at a fixed point at point K, while in the transfer test, experimenter threw the ball randomly at point E to any point within the green area (as shown in Fig. 1), which increased the difficulty of hitting the ball.

#### 2.3.6 Evaluation indicators

Batting accuracy: The test subject stands at point T, the experimenter threw the ball at point K for the pre-test and retention test, and at point E for the transfer test. Two camera positions, C1 and C2, are set up to capture the action. On the right side of the field, opposite to the subject, three scoring areas have been marked out. Hitting the ball into areas 1, 2, and 3 will respectively score 1, 2, and 3 points. Failure to hit the ball into any of these areas will result in zero points (as shown in Fig. 1).

Action scores: The video of each subject's batting action was randomly edited into independent units, and three independent raters independently assessed the batting action postures in accordance with the rules and the requirements of the standardized actions, and took the average scores of the three, with higher scores indicating a more standardized action of the subject. The total score for the action was 100 points. 80 points allocated for movement completeness, which included 10 points for preparation posture (2 points per entry, 5 entries), 48 points for the backswing and swing posture, 10 points for lowering posture (2 points per entry, 5 entries) and 12 points for follow-through posture (3 points per entry, 4 entries). The remaining 20 points were dedicated to movement fluency, with the ratio of completeness points to fluency points being 1:4 (rounded up to the nearest whole number).

Number of knowledge mastery: The number of explicit knowledges was 15, while the number of analogical knowledges was 6. Each number contributed 1 point. The amount of knowledge mastery was assessed by three independent raters, and their scores were averaged.

#### 2.3.7 Experimental equipment and site

The venue was a children's short-net court measuring 13.4 m × 6.1 m, 13 tennis racquets of the same model (25″) and 100 new tennis balls (orange balls), two video cameras.

#### 2.3.8 Data acquisition and analysis

One camera was placed on the right side of the subject at a height of about 1.4 m, which was convenient for clearly capturing the complete movements of the subject; the other camera was placed on the other side of the net, outside the sideline, at a height of about 0.3 m, which was convenient for accurately recording the scores.

The statistical software SPSS 25.0 was used for data processing, with a significant level of α = 0.05.

## 3 Results

### 3.1 Batting accuracy

Descriptive statistics were performed on batting accuracy in the retention test and the transfer test. The mean value of batting accuracy in the retention test was 15.23 with a standard deviation of 4.58 for the explicit-analogical group; the mean value of the analogical-explicit group was 21.85 with a standard deviation of 3.51; and the mean value of the alternation group was 17.69 with a standard deviation of 2.98. The mean value of batting accuracy for the explicit-analogical group of the transfer test was 12.38 with a standard deviation of 4.82; the mean value of the analogical-explicit group was 20.23 with a standard deviation of 3.19; and for the alternation group, the mean was 14.69 with a standard deviation of 4.25 (as shown in Table 2).

**Table 2:** Descriptive statistics of test results.

		Batting accuracy	Action Scores			Number of knowledge mastery
			Movement Integrity	Movement fluidity	Total scores	
Pre-test	1	5.15 ± 1.21	19.63 ± 1.16	4.91 ± 0.29	24.54 ± 1.45	0
	2	5.23 ± 0.93	19.75 ± 0.89	4.94 ± 0.22	24.69 ± 1.11	0
	3	5.15 ± 0.89	19.26 ± 1.33	4.82 ± 0.33	24.08 ± 1.66	0
Retention test	1	15.23 ± 4.58	55.32 ± 4.72	13.83 ± 1.18	69.15 ± 5.89	12.46 ± 1.81
	2	21.85 ± 3.51	59.63 ± 4.67	14.91 ± 1.17	74.54 ± 5.83	17.38 ± 1.33
	3	17.69 ± 2.98	55.38 ± 5.76	13.85 ± 1.44	69.23 ± 7.20	15.23 ± 1.17
Transfer test	1	12.38 ± 4.82	57.23 ± 5.33	14.31 ± 1.33	71.54 ± 6.67	11.85 ± 1.52
	2	20.23 ± 3.19	65.42 ± 4.12	16.35 ± 1.03	81.77 ± 5.15	17.62 ± 1.04
	3	14.69 ± 4.25	59.20 ± 4.36	15.15 ± 1.43	74.00 ± 5.45	14.77 ± 1.24

As shown in Fig. 2, a one-way ANOVA was conducted on batting accuracy in the retention test and the transfer test, and the between-group F = 10.324, p < 0.01, for the three groups in the retention test was highly significant; in the transfer test, the between-group F = 12.311, p < 0.01, and the between-group difference was highly significant. A post hoc test found that in the retention test, there was a significant difference between the three groups (p < 0.001; p = 0.008), whereas there was no significant difference between the analogical-explicit group and alternation group (p = 0.103). In the transfer test, there was a significant difference between the three groups (p < 0.001; p = 0.002), while there was no significant difference between the explicit-analogical and alternation groups (p = 0.164).

**Fig. 2:** Analysis of differences in batting accuracy. (Note: ∗p < 0.05, ∗∗p < 0.01, same below).

### 3.2 Action scores

Descriptive statistics were performed on the action scores of the retention and transfer tests. The mean of the action scores of the explicit-analogical group in the retention test was 69.15 with a standard deviation of 5.9, the mean of the analogical-explicit group was 74.54 with a standard deviation of 5.84, and the mean of the alternation group was 69.23 with a standard deviation of 7.20. The mean value of the action scores for the explicit-analogical group of the transfer test was 71.54 with a standard deviation of 6.67, the mean value of the analogical-explicit group was 81.77 with a standard deviation of 5.15, and the mean for the alternation group was 74 with a standard deviation of 5.45 (as shown in Table 2).

As shown in Fig. 3, a one-way ANOVA was conducted on the movement scores of the retention test and the transfer test, with no significant between-group difference of F = 3.077, p > 0.05 for the three groups in the retention test, and a highly significant between-group difference of F = 11.051, p < 0.01 for the three groups in the transfer test. A post-hoc test revealed that in the transfer test, the analogical-explicit group differed significantly from both the explicit-analogical and alternation groups (p < 0.001; p = 0.002), whereas the explicit-analogical group did not differ significantly from the alternation group (p = 0.286). This suggests that the techniques of the three groups were unaffected in the retention test without increasing the difficulty, whereas when the difficulty was increased for the transfer test, analogical-explicit group were significantly better than the other two groups.

**Fig. 3:** Analysis of differences in action scores.

### 3.3 Number of knowledge mastery

Descriptive statistics were performed on the number of knowledge mastery in the retention and transfer tests. The mean value of the number of knowledge mastery of the explicit-analogical group in the retention test was 12.46 with a standard deviation of 1.81, the mean value of the analogical-explicit group was 17.38 with a standard deviation of 1.32, and the mean value of the alternation group was 15.23 with a standard deviation of 1.17. The mean value of the number of knowledge mastery of the explicit-analogical group in the transfer test was 11.85 with a standard deviation of 1.52, the mean value of the analogical-explicit group was 17.62 with a standard deviation of 1.04, and the mean value of the alternation group was 14.77 with a standard deviation of 1.24. The mean value of the number of knowledge mastery in the explicit-analogical group was 11.85 with a standard deviation of 1.52, the mean value of the analogical-explicit group was 17.62 with a standard deviation of 1.04, and the mean value of the alternation group was 14.77 with a standard deviation of 1.24(as shown in Table 2).

As shown in Fig. 4, the number of knowledge mastery in the pre-test was zero, indicating that none of the subjects had mastered the essentials of the two-handed backhand stroke. A one-way ANOVA was conducted to analyze the number of knowledges acquired in the retention test and the transfer test. The difference was highly significant in the retention test, with the between-groups of the three groups F = 37.205, p < 0.01. The difference was highly significant in the transfer test with the between-groups of the three groups F = 65.922, p < 0.01. A post hoc test found that in the retention test, there was a significant difference between the three groups (p < 0.001; p = 0.001), as well as between the explicit-analogical group and the alternation group (p < 0.001). In the transfer test, there was a significant difference between all three groups two by two (p < 0.001).

**Fig. 4:** Analysis of differences in number of knowledge mastery.

## 4 Discussion

The results of the study indicate a significant main effect of learning style on subjects' performance. Specifically, in the retention test, the group that learned through analogical-explicit group performed better than the explicit-analogical and alternation groups. Dual encoding divides long-term memory into the representational and verbal systems, which are both independent of and interconnected with each other and are involved in information processing for motor skill learning [19]. In the analogical-explicit group, analogical learning encodes information in the form of representations. The metaphor of forehand striking action has “examples” and “prototypes” in practice. Based on the similarity between the two, it forms a concrete, vivid and real perceptual image in the human brain through the sensory effect, which reflects the forehand striking action from the overall perspective, which is easy for learners to memorize and helps to build up the overall sports image. Moreover, the use of metaphors helps to reduce working memory load while expanding its information capacity, allowing for better processing of explicit learning instructions. Learners can use explicit knowledge to semantically characterize the kinematic features of the forehand stroke, such as form and trajectory, providing references for feedback and enabling learners to purposefully improve their strokes. During this process, precise explicit learning gradually solidifies analogical knowledge, while generalized analogical learning visualizes explicit knowledge. This promotes the absorption and assimilation of knowledge as the two types of knowledge dynamically integrate with each other, forming a synthesis. As a result, learners find it easier to grasp the key points of the forehand stroke, develop proper movement posture, and enhance stroke accuracy. Beginners often struggle to understand the terminology used in explicit learning. However, analogical learning, with its metaphorical terminology, is more accessible and easier for them to comprehend and learn [20]. By combining analogical learning with subsequent explicit learning, beginners can quickly establish a clearer and more precise motor representation. This, in turn, helps them establish correct self-diagnostic evaluation criteria and accelerates the process of translating motor representation into the concept of movement. Consequently, the internal feedback abilities of practitioners improve, leading to enhanced motor skills. By improving the practitioner's internal information feedback ability, overall learning of motor skills is further enhanced.

The 15 explicit knowledges that the learners in the explicit-analogical group received first was specific, but it was more difficult to process numerous pieces of information in a short period of time, affecting the mastery of movement essentials, which in turn affected the improvement of movement postures and batting accuracy. On the other hand, the learners in the analogical-explicit group received 6 metaphors that lacked the feature of the kinematics of the movement. In contrast, beginner learners in the child group excel at imitation, enabling them to quickly master the technical movement. Once a general framework for the technical movement is established, the explicit knowledge can be utilized to correct the finer details, thereby refining the technical movement and enhancing batting accuracy. The learners in the alternation group, who simultaneously learned explicit and analogical knowledge, faced challenges due to their limited comprehension and logical analysis skills as beginners. Consequently, they struggled to absorb a greater volume of knowledge and often forgot the technical movement concepts. This resulted in the breakdown of movement integrity and standardization, ultimately impacting batting accuracy.

According to SCHMIDT's schema theory, the transfer test assesses general movement procedures, which are abstract representations of a particular type of movement stored in memory [21]. These procedures encompass the fundamental characteristics and parameters of a skill, such as relative timing, relative force, and the sequence of movement components. During the transfer test, the analogical-explicit group outperformed the explicit-analogical group and the alternation group. This suggests that this combination may be beneficial for the development of general motor programs in novice children. However, further exploration is needed to fully understand the underlying reasons for this observation [22].

Yu et al. explored the role of synergistic mechanisms of analogical and explicit learning in adolescent tennis beginners of different ages and concluded that college students had better performance with alternating analogical and explicit learning, whereas junior high school students had better performance with analogical-explicit learning [23]. However, due to the limited cognitive processing ability and working memory capacity of beginner children, the large amount of explicit information received by the explicit-analogical group and the alternation group overloads their working memory. As a result, they struggled to switch between memorized instructions and skill operations, leading to confusion and a decrease in the efficiency of learning movement essentials and postures. One solution to this problem is to use the way of analogies to demonstrate and guide beginners during initial practice. This approach helps them establish a framework for the movement and master the key components of the technical movement. Afterwards, they can be guided to focus on strengthening the details of the movement through language and other means. By reducing the amount of information that learners need to process, the six instructions received by the analogical-explicit group in the first module alleviated the working memory load. Additionally, the analogies vividly describe the movement of forehand strokes using familiar experiences, making it easier and more enjoyable for learners to understand and accept. The intuitive and holistic nature of the analogies helps beginners construct a more complete and deeper understanding of the movement, ultimately facilitating the development of a holistic picture of the movement. In Module 2, the explicit learning guide provides detailed descriptions of the rhythm, sequence, and other fixed characteristics and parameters necessary for accomplishing the forehand stroke. This approach not only avoids negative transfer caused by analogical learning and the formation of incorrect movements, but also reduces teaching blindness. As a result, the learning process is accelerated, and the standardization of the movement is promoted.

The combination of analogical and explicit learning as a teaching method offers several advantages. Firstly, it helps learners connect new knowledge with their existing cognitive structure by presenting instructions in a clear and familiar manner. This facilitates a high degree of generalization, particularly in the context of the forehand stroke. By integrating the new knowledge into their existing cognitive structure, learners can better understand the essentials of the forehand technical movement and promote positive transfer of this skill. The teaching approach follows a logical progression from easy to difficult and from simple to complex. This enables beginners to transition from a stage of rough mastery to one of consolidation and improvement, allowing them to quickly master the technical movements. To accommodate the thinking characteristics of beginners and reduce their difficulties in comprehending abstract concepts, it is important to organize the teaching in a manner that aligns with their cognitive abilities. During the transfer test, the group utilizing the analogical-explicit learning method outperformed the groups using the explicit-analogical and alternating methods. This indicates that the analogical-explicit method is more effective in establishing and forming general motor programs in beginner children. However, further research is needed to fully understand the underlying mechanisms behind this result.

Most of the current research focuses on the independent effects of analogical and explicit learning, while this study explores the synergistic effect between the two, combining them by using a one-factor experiment. In addition, most scholars focus more on adolescents and adults as the research object, while this paper takes children as the research object, which broadens the research object group and provides a theoretical basis for the development of children's tennis. There are two main limitations of this study. First, the experimental period is short. The subjects are all elementary school students, whose use of summer vacation to learn tennis, making it difficult to conduct a long experiment; the second is the limitation of the experimental design. Due to the experimental period, there was not enough time to conduct the retention test at intervals of a few days after the end of the practice, and it was difficult to control the subjects not to practice tennis during this period of time, so the retention test was conducted sometime after the end of the training. The limitations of the study may have affected the generalization of the results and conclusions, but the exact impact is uncertain. In the future, the mechanisms by which analogical and explicit learning affect the acquisition of tennis skills in children's beginners and the mechanisms by which the brain processes verbal and figurative coding processing in the process could be explored in depth. The effects of different combinations of the two in other open motor skill and closed motor skill and the optimal combination of the two can be further investigated for different groups.

## 5 Conclusion

This study investigated the different synergistic effects of analogical learning and explicit learning in the learning of motor skills by beginner children's tennis players, and the results confirmed the expected hypothesis that the different combinations of analogical learning and explicit learning are one of the important factors affecting the learning performance of motor skills, which also applies to the learning of sensory skills and other similar skills. Studying the synergistic effect of analogical learning and explicit learning is beneficial to improving the learning effect, promoting skill mastery, and enriching the theoretical and practical results of motor skills. However, analogical learning relies more on existing experience and is more subjective, and analogical learning is conducive to the construction of movement frames but is not conducive to the reinforcement of movement details, so it should be considered comprehensively in actual teaching to bring the synergistic effect into play to achieve the best results. The results of the study showed that the analogical-explicit group performed better than the explicit-analogical group and the alternation group in the learning and mastery of children's beginner tennis skills. This reveals that in teaching and training of children's tennis, coaches should pay special attention to teaching analogies and giving more demonstrations and explanations to improve teaching efficiency and enhance children's physical fitness. Researchers should further explore the influence mechanism of analogical learning and explicit learning on the skill mastery of beginners, so as to provide a theoretical basis for the practical application of the two.

## Funding sources

This work was supported by the Department of Higher Education of the Ministry of Education of China and Beijing Zhixing Lingdang Technology Co [Grant number: CICA2020103]; Beijing Academy of Educational Sciences [Grant number: 220900239235815].

## Data availability statement

All data generated or analyzed during this study are included in this article and supp. material in article.

## CRediT authorship contribution statement

**Jiyan Xu:** Writing – original draft, Validation, Methodology, Data curation. **Weiwei Xu:** Writing – review & editing, Methodology, Conceptualization. **Mengjiao Sang:** Writing – review & editing, Supervision.

## Declaration of competing interest

The authors declare that they have no known competing financial interests or personal relationships that could have appeared to influence the work reported in this paper.
